# Analysis of Related Factors of Mother-to-Child Transmission of AIDS and Evaluation of Measures to Prevent Mother-to-Child Transmission

**DOI:** 10.1155/2022/3190370

**Published:** 2022-01-05

**Authors:** Yuhuan Liu, Yulan Zhang, Lin Pang

**Affiliations:** ^1^Pediatric Department, Beijing Ditan Hospital Affiliated to Capital Medical University, Beijing 100015, China; ^2^Hospital Management, People's Hospital of Deyang City, Deyang, Sichuan 618000, China

## Abstract

AIDS is still a major public health facing the world. With the implementation of AIDS prevention projects and the continuous maturity of technology, more and more HIV-positive women choose to have children. However, the children born to these women are a special group. Exposure to HIV and antiviral drugs during the fetal period can increase the success rate of children's elimination of the mother, which is worthy of attention and research. This article focuses on the analysis of the related factors of mother-to-child transmission of AIDS and the evaluation of mother-to-child blocking measures, using the method of field research to conduct experiments on AIDS patients in this city who are pregnant and provide them with antidrug treatment and some barrier measures. Then, the mother-to-child transmission rate was recorded, and the experimental results showed that the antidrug treatment plan is related to mother-to-child transmission. After antidrug treatment, the transmission rate of single-drug treatment is reduced by 5%, and the transmission rate of combined drug treatment is reduced by 10%. It can be seen from this that antidrug treatment is an effective measure to block mothers and babies.

## 1. Introductions

Mother-to-child transmission of HIV (MTCT) is one of the main causes of the HIV epidemic, accounting for approximately 9% of new infections worldwide [1, 2]. Mother-to-child transmission of HIV is the infection of HIV carriers through childbirth, pregnancy, childbirth, or breastfeeding after being infected with the virus [3, 4]. Without treatment, babies born to HIV-positive women are 15-30% more likely to be infected with the virus during pregnancy or childbirth and 5-15% more likely to contract the virus through breastfeeding [5, 6]. Through breastfeeding, the HIV infection rate is as high as 36.4% [7, 8].

For the study of mother-to-child transmission of AIDS, some researchers have evaluated the cost of providing services to prevent mother-to-child transmission of HIV/AIDS (PMTCT) under different epidemic (high and low) and socioeconomic (urban and rural) backgrounds, using microcost calculation methods to identify, measure, and evaluate the resources used to provide comprehensive PMTCT services. The results show that the average cost per pregnant-infant (PPY) pair in the high HIV city ranges from 6,280 ETB (US$319) to 21,620 ETB (US$1,099), etc. [9]. There are also researchers who evaluated the effectiveness of the city government-led all-round multilevel cooperation platform model in blocking mother-to-child transmission of AIDS. The method was to select 339 136 newly diagnosed pregnant women from health care institutions at all levels and divide them into two groups: the first group is composed of unresearched subjects, and the second group is the control group; the two groups are AIDS regular health education and AIDS testing; adopt the government-led all-round multilevel cooperation platform work model to intervene in the observation group and compare the proportion of pregnant women tested for HIV antibody, HIV antibody positive rate, and pregnancy failure rate [10]. There are also researchers aiming at blocking mother-to-child transmission with combined drug therapy, and they selected 150 cases of human immunodeficiency virus- (HIV-) positive pregnant women in 2014 and divided them into experimental groups based on positive antibodies and intervention during pregnancy (detected before 14 weeks of gestation); 75 cases were compared with the control group (found after 14 weeks of gestation) to compare the levels of serum inflammatory markers (TNF-*α*, hs-CRP, and Ang-II), viral load, and infant HIV infection between the two groups and found to have obvious representational meaning [11]. There are also investigators aiming at the prevention of mother-to-child transmission of human immunodeficiency virus (HIV). The results of HIV-infected women recruited in a prospective cohort study of international maternity, gynecology, and pediatric adolescent AIDS clinical trials (plan P1025) showed that in 1,857, there were 12 cases of mother-to-child transmission of HIV among live-born newborns, and for every 100 live births among women infected with HIV, there were 0.65 cases (95% confidence interval 0.33-1.13) [12]. In summary, the world pays more attention to AIDS, and there are more studies on the factors of AIDS transmission and measures to block the transmission of AIDS, but there are few results in the study of mother-to-child transmission alone.

This article conducts research on the analysis of related factors of mother-to-child transmission of AIDS and the evaluation of measures to prevent mother-to-child transmission. On the basis of relevant literature data, we understand some theories of mother-to-child transmission of AIDS and then analyze some influencing factors of mother-to-child transmission of AIDS. Using field research methods, experimental verification of AIDS transmission factors and barrier measures is carried out, and relevant conclusions are drawn through experimental results.

## 2. Research on Related Factors of Mother-to-Child Transmission of AIDS and Measures to Prevent Mother-to-Child Transmission

### 2.1. Mother-to-Child Transmission of AIDS

#### 2.1.1. Intrauterine Transmission

HIV infects the fetus through the placental barrier at any time during pregnancy, leading to mother-to-child transmission.

#### 2.1.2. Spread during Childbirth

If there is HIV in the mother's reproductive tract and the baby directly contacts the mother's blood, the secretions in the birth canal will cause infection, leading to the amount of virus in the fetus in the mother's birth canal. Obstetric trauma surgery, such as episiotomy, forceps, and suction delivery, increases the risk of mother-to-child transmission.

#### 2.1.3. Postpartum Breastfeeding Spread

The HIV content in breast milk is high. Studies have shown that the risk of mother-to-child transmission from breastfeeding is about 10% to 20%. The more you breastfeed, the higher the risk of mother-to-child transmission. In addition, breastfeeding can damage the inner wall of the baby's digestive tract, increasing the risk of infection.

### 2.2. Measures to Block Mothers and Infants

1. Pay attention to the use or even use of appropriate drugs before delivery to minimize the virus in pregnant women, and use drugs to reduce it to an undetectable state
2. Caesarean section is recommended during childbirth, because it can prevent damage to the baby's skin and mucous membrane. This shortens the delivery process and reduces the torture of the patient during the delivery process. At the same time, it prevents child from contracting the virus
3. After giving birth to a child, try to avoid breastfeeding. At the same time, avoid contacting the patient's blood and body fluids with the child, so as to have a preventive effect

### 2.3. Influencing Factors of Mother-to-Child Transmission

#### 2.3.1. Sociological Factors

The influence of social factors on mother-to-child transmission of AIDS is mainly affected by many aspects, including socioeconomic impact, sociodemographic impact, and knowledge of HIV/AIDS. Therefore, the higher the female Hrv infection rate, the greater the possibility of mother-to-child transmission. Whether personal education and living standards affect the mother-to-child transmission of Hrv virus is mostly a combination of multiple factors.

#### 2.3.2. Biological Factors

Biological factors are directly related to pregnant women from pregnancy to delivery and lactation, such as viral factors and placental factors. Studies have shown that the main cause of vertical transmission is the condition of pregnant women, and the number of viruses directly determines the possibility of vertical transmission. The higher the viral load, the greater the possibility of HIV transmission from mother to child. The lower the vitamin a content in the mother's body, the more likely the mother is to be infected with HIV. The medical history of the pregnant woman (sexually transmitted diseases, hepatitis c, chorioamnionitis, etc.) can also affect the possibility of mother-to-child transmission.

### 2.4. Data Processing

Logistic regression analysis is a generalized model of linear regression analysis, which is often used in fields related to data analysis such as disease diagnosis and economic forecasting. There is regression in the definition, but it is essentially linear regression. If the linear regression output is continuous and cannot limit the range of values, the linear sum of the attributes can be used to match the attributes with the results. A function map that uses the *g*(*z*) function to calculate continuous values and assigns them to 0 or 1 has been added. Regression is a classification algorithm, mainly used for two classification problems. However, unlike linear regression, logistic regression compresses the output range from 0 to 1. This eliminates the influence of particularly strong variables in the model. The function (or sigmoid function) form is as follows:

(1) $$\begin{array}{c} g\left(z\right)=\frac{1}{1+e^{-z}}, \end{array}$$

where *e* is the parameter.

For a given *n* features, let the conditional probability of the observation sample *y* relative to the event occurrence factor *x* be *p*(*y* = 1 | *x*), expressed by the logistic function as follows:

(2) $$\begin{array}{c} p\left(y=1\left|x\right.\right)=\pi \left(x\right)=\frac{1}{1+e^{-g\left(x\right)}}, \end{array}$$

## 3. Evaluation Experiment on Factors Related to Mother-to-Child Transmission of AIDS and Measures to Prevent Mother-to-Child Transmission

### 3.1. Research Methods

From 2019 to 2020, the survey site will conduct recruitment (baseline survey) and track data collection from birth to 19 months. A total of 135 cases were collected. All pregnant women and children living with HIV in the study area were referred to the study. We will collect and obtain informed consent and important and other relevant information as early as possible during pregnancy; due to the limited number of research topics, we will try to exclude all pregnant women infected with HIV and recruit a research team to collect information, including relevant obstetric information, especially delivery methods, working hours, obstetric trauma, and other relevant information until delivery. According to different delivery methods, women and newborns infected with HIV are divided into exposure group and control group. Regular/postpartum follow-ups were conducted at 2, 4, 7, 8, 14, and 19 months, respectively, to understand the birth survival rate and HIV infection status. Basic research and follow-up research are done by local trained researchers. The study tested feeding and childbirth as confounding factors and excluded researchers who were not artificially fed and also excluded embryos born from twins.

### 3.2. Inclusion Criteria of Experimenters

1. Pregnant women are between 20 and 40 years old at childbirth
2. In addition to receiving HIV antiviral during pregnancy, no other drugs were used
3. All newborns received standardized, active, and passive combined immunization throughout the whole course and followed up until the age of 2 to 19 months

### 3.3. Establishment of the Database

#### 3.3.1. Patient's Information

*(1) Antidrug Program*. Patients on the azt+nvp regimen can receive 8 to 108 doses, *m* = 50 doses. Patients on the azt+3tc+nvp/efv regimen received 1-280 doses, *m* = 71.5 doses. Seven mothers refused to take HIV, of which three refused to take it by themselves, four pregnant women with HIV refused to take it, and the mother refused to take it for the child. The refusal rate was about 4.2% (7/168). In 7 cases of pregnancy, one dose was missed, but one dose was missed (complete missed dose rate is less than 5%), at least 2 times, up to 4 times (forgot to take rate less than 5%), and 4 cases after delivery of newborns forgot to take medication at home. One case missed 3 times after taking 7 days each time (forgetting taking rate = 10.7%), 1 case was stopped after 7 days, and 2 cases took the number of days after 42 days (1 case missed one time, and 1 case missed taking medicine), 2 doses; all missed doses are less than 5%.

*(1) Health Status*. There is 1 case of liver dysfunction. Hemoglobin surveillance: the prevalence of anemia in pregnancy and children infected with HIV is approximately 47.8% (65/136). The number of bits is set to 110 g/dl, pz = 103 g/dl, the minimum is set to 11 g/dl, and the maximum is set to 155 g/dl. Among them, 7 cases were below 90 g/dl and 158 cases were 90-110 g/d. CD4 monitoring: the better range is 2~1178 cells/ml, and the median value is 345 cells/ml. Among them, less than 50 cells/ml have 34 packs, 250-350 cells/ml have 35 packs, and more than 50 cells/ml have 67 cases.

#### 3.3.2. Children's Information

A 12-month-old baby uses fingertip venous blood for prescreening with Abbott's rapid test kit. The test results showed that HIV-infected persons were negative and were excluded from HIV infection. The preliminary test was HIV-positive. Completing blood collection at 19 months of age requires rescreening and confirmation. This experiment mainly used the Abbott rapid test strip and enzyme-linked immunosorbent assay (ELISA). If it is negative, HIV infection can be ruled out. If all the results are positive, or the test results are invalid, please use the wb test of Singapore Asia Pacific Reagents. If the wb test is negative, then it is positive, the wb is diagnosed as positive, and there is HIV infection.

### 3.4. Statistical Methods

The database is a statistical analysis and calculation using the SPSS 200 software. Observed data is usually expressed in terms of mean ± standard deviation. A pair of *t*-tests was used to observe the effect of patients on the results of the test before and after treatment. The differences between the groups were compared by analysis of variance. *P* < 0.05 indicates that the difference is statistically significant, and *P* < 0.01 indicates that the deviation is statistically significant. Counting data is expressed as a percentage, and the comparison of percentages is tested by card method. If the theoretical frequency is less than 5, you can use Fisher's precise method to test.

## 4. Analysis of Experimental Results

### 4.1. Analysis of General Patient Data

By sorting out the education level of the patients and the quality of their compliance with the doctors during the experiment, the relevant data are shown in Table 1.

It can be seen from Figure 1 that most of the experimenters have junior high school education, 51 with junior high school education, and 70 with high school education. It can be seen that the cultural background is not relevant.

### 4.2. The Relationship between Mother-to-Child Transmission of AIDS and Mother's Infection Status

The biological characteristics such as CD4+ T lymphocyte count and HIV viral load of infected pregnant and lying-in women were stratified and analyzed. The relevant data are shown in Table 2.

As can be seen from Figure 2, the higher the detection of the virus, the higher the probability of mother-to-child transmission. Therefore, the barrier to mother-to-child transmission is to minimize the virus in the body, which can reduce the transmission rate.

### 4.3. The Impact of Antiviral Treatment on Mother-to-Child Transmission of AIDS

The antiviral treatment characteristics of HIV-infected pregnant women, such as the antiviral treatment plan, the starting period of medication, and the degree of standardized medication, were stratified and analyzed. The relevant data are shown in Table 3.

It can be seen from Figure 3 that mother-to-child transmission of AIDS is related to antidrug treatment during pregnancy. The transmission rate of unused antidrug is obviously higher than the used transmission rate, and the antidrug effect of a single drug is not very good, only reduced 5%; the effect of combination therapy is the best, reducing by 10%.

### 4.4. The Relationship between Pregnancy and Childbirth Complications and Mother-to-Child Transmission of AIDS

The characteristics of pregnancy and childbirth complications such as HIV-infected pregnant women with hepatitis, vaginitis, and sexually transmitted diseases were stratified and analyzed. The relevant data are shown in Table 4.

It can be seen from Figure 4 that the transmission rate of patients with hepatitis is higher than that of the other two diseases. The transmission rate of patients with hepatitis is 11.9%, while the transmission rate of patients with vaginitis is 6.9%.

### 4.5. Related Suggestions

1. Strengthen health education, detect infected persons early, strengthen follow-up of positive women, and reduce unwanted pregnancies

Raise the people's awareness of the AIDS epidemic and strengthen control. Since the infected are mainly farmers, it is necessary to strengthen the knowledge of AIDS prevention and control of the floating population in accordance with national customs, promote responsible sexual behavior or avoid high-risk behaviors, and postpone early sexual activities. The use of condoms in age, abstinence, or extramarital sex should be postponed and encouraged.

(2) Further improve the maternal and child health care network, cooperate with multiple departments, improve the early pregnancy detection rate and the quality of pregnancy and childbirth health care, and increase the anti-HIV drug use rate and drug testing

Rural traffic is inconvenient, and the network is not perfect. It is unable to provide services for public maternity and child health projects. The city's maternity and child health resources are reasonably allocated for AIDS testing, maternity health care, and childbirth services. This not only reduces the financial burden of pregnant women's families but also helps to continue AIDS screening and counseling services as early as possible in the first semester or early. For contraception, use domestic rapid test strips for the first test, and use the first test or imported rapid test strips for a second test immediately after the test is positive. In the second test, antiviral drugs were given immediately after the test was positive.

## 5. Conclusions

This article focuses on the analysis of factors related to mother-to-child transmission of AIDS and the evaluation of measures to prevent mother-to-child transmission. Through experiments on pregnant women with AIDS admitted to hospitals in this city, the results of the experiments show that antidrug treatment is aimed at mother-to-child transmission. The effective measure to block is to reduce the transmission rate by 5% when the drug is administered alone and by 10% when used in combination with drugs, but the transmission rate of the mode of delivery needs certain research. There are still some shortcomings in the research process of this article, mainly manifested in the lack of research depth.

## Figures and Tables

**Figure 1:** General patient data analysis.

**Figure 2:** The relationship between mother-to-child transmission of AIDS and mother's infection status.

**Figure 3:** The impact of antiviral treatment on mother-to-child transmission of AIDS.

**Figure 4:** The relationship between pregnancy and childbirth complications and mother-to-child transmission of AIDS.

**Table 1:** General patient data analysis.

	Exposure group	Control group
Junior high school culture	21	30
High school culture	21	49
University culture	1	7

**Table 2:** The relationship between mother-to-child transmission of AIDS and mother's infection status.

	Exposure group	Control group
CD4+ T lymphocyte count	6.5	8.1
	6.4	6.2

Viral load	9.5	4.3
	14.8	10.9

**Table 3:** The impact of antiviral treatment on mother-to-child transmission of AIDS.

	Exposure group	Control group
No medication	15.5	8.5
Single plan	10.3	7.5
Joint program	2.6	4.7

**Table 4:** The relationship between pregnancy and childbirth complications and mother-to-child transmission of AIDS.

	Exposure group	Control group
Hepatitis	11.1	9.4
Vaginitis	6.9	5.3
Sexually transmitted diseases	0	7.5

## Data Availability

The data underlying the results presented in the study are available within the manuscript.
